# HNRNPA2B1 Demonstrates Diagnostic and Prognostic Values Based on Pan-Cancer Analyses

**DOI:** 10.1155/2022/9867660

**Published:** 2022-04-27

**Authors:** Chaoyang Chen, Lipeng Huang, Qingyu Sun, Zhichen Yu, Xiaoyan Wang, Liang Bu

**Affiliations:** Department of Thoracic Surgery, Xiamen University Institute of Chest and Lung Disease, Xiang'an Hospital of Xiamen University, China

## Abstract

Some studies have suggested heterogeneous nuclear ribonucleoprotein A2/B1 (HNRNPA2B1) to be a promoter in cancer development. Nonetheless, no detailed pan-cancer investigation has been reported. Thus, this study explored the possible oncogenic role of HNRNPA2B1, such as its expression levels, gene alteration, protein–protein interaction network, immune infiltration, and prognostic value in different cancer types using The Cancer Genome Atlas web platform. Many types of cancer exhibit HNRNPA2B1 overexpression, which is notably associated with poor prognosis. We also found that HNRNPA2B1 with different methylation levels causes a varied prognosis in lung adenocarcinoma (LUAD). It is noteworthy that HNRNPA2B1 levels are connected with cancer-associated fibroblasts in cancers, such as adrenocortical carcinoma, LUAD, and stomach adenocarcinoma. In addition, HNRNPA2B1 participates in the spliceosome- and cell cycle-associated pathways. Finally, HNRNPA2B1 is highly valued in the diagnosis of LUAD, lung squamous cell carcinoma, breast invasive carcinoma, esophageal carcinoma, and liver hepatocellular carcinoma. This systematic study highlighted the role of HNRNPA2B1 in pan-cancer progression.

## 1. Introduction

Cancer is one of the leading causes of death worldwide. It is also a predominant burden to elevated life expectancy [1]. Recent studies have revealed that the rates of cancer incidence and death are continuously growing in most developing countries. Because cancer incidence is complex and varied, exploring the association among genes, prognosis, and signaling pathways in different cancer types was difficult. However, with the emergence of public databases such as The Cancer Genome Atlas (TCGA) [2] and Gene Expression Omnibus [3], the analysis of genes through pan-cancer investigations has become popular [4–6]. We also used TCGA database to obtain the data on different tumors for this pan-cancer study.

Heterogeneous nuclear ribonucleoprotein A2/B1 (HNRNPA2B1), as an N6-methyladenosine (m6a) reader, exhibits key effects on RNA splicing [7], antiviral immunity [8], miRNA biogenesis [9], etc. Recently, it has been reported that HNRNPA2B1 is involved in the recognition of pathogenic DNA and the elaboration of the innate immune response [10]. Previously, research data revealed that HNRNPA2B1 stimulates the development of cancer, such as pancreatic cancer and non-small-cell lung cancer (NSCLC) [9, 11]. Surprisingly, we found that inhibiting HNRNPA2B1 expression can reduce the proliferation rate of lung cancer cells [12]. According to some bioinformatics analyses, HNRNPA2B1 is associated with other m6A regulators in various cancers. HNRNPA2B1 is a new prognosis biomarker for patients with ovarian cancer (OC) [13]. Both ALKBH5 and HNRNPA2B1 were found to be significantly associated with poor outcomes in patients with TP53-mutant NSCLC [14]. Increased HNRNPA2B1, VIRMA, and IGF2BP3 were associated with poor prognosis in esophageal cancer [15]. Recently, it has been indicated that HNRNPA2B1 serves as a long noncoding RNA- (lncRNA-) or miRNA-binding protein. MIR100HG interacts with HNRNPA2B1 to regulate TCF7L2 mRNA stability in colorectal cancer [16]. With the aid of HNRNPA2B1, the pri-Let-7b processing increased the mature Let-7b level to suppress the Notch signaling in osimertinib treatment [17]. However, the association between abnormal HNRNPA2B1 levels and tumor prognosis and immunity in pan-cancer has not been reported.

Using TCGA database, this study completed a pan-cancer study of HNRNPA2B1. We also evaluated gene expression levels, survival rates, methylation status, changes in protein phosphorylation, immune cell infiltration, and related signaling pathways to see if HNRNPA2B1 could play a role in pan-cancer prognosis.

## 2. Materials and Methods

### 2.1. Evaluation of Gene Expression Levels in Pan-Cancer

HNRNPA2B1 expression levels were determined using the “Gene_DE” module in the TIMER (http://timer.cistrome.org/) web platform, while HNRNPA2B1 levels in the tumor and corresponding normal tissues were determined via TCGA. All the raw data were standardized using log2 TPM transformation. HNRNPA2B1 levels in tumors and adjacent normal tissue samples were also determined using GEPIA2 (http://gepia2.cancer-pku.cn/#general) [18].

### 2.2. Evaluation of Survival Prognosis in Different Cancer Types

The prognostic values of HNRNPA2B1 were measured using the Kaplan–Meier method with significance set at *P* < 0.05, and the significance charts of overall survival (OS) in pan-cancers were obtained.

### 2.3. Investigation of Mutation and Methylation Status of HNRNPA2B1 and Its Applications in Prognosis

cBioPortal (https://www.cbioportal.org/) was used to determine the mutation status of HNRNPA2B1 [19]. HNRNPA2B1 genomic profiles with *z*-score thresholds of 1.5 were used. Genetic mutations in HNRNPA2B1 and their association with OS were assessed to determine its prognostic value. HNRNPA2B1 methylation data were obtained from the cBioPortal. The relationship between HNRNPA2B1 expression levels and copy number was investigated. Furthermore, the prognostic values of HNRNPA2B1 methylation status in lung adenocarcinoma (LUAD) were investigated using the MethSurv web tool, which is a useful tool for providing survival studies based on DNA methylation biomarkers through TCGA database.

### 2.4. Evaluation of the Infiltration of Immune Cells

The types of immune cells and their corresponding infiltration data were obtained from the TIMER Database's Immune-Gene module. The changes in immune cell infiltration in the high/low HNRNPA2B1 groups were measured, and the relationship between immune cells and HNRNPA2B1 was investigated. The *P* values and partial correlation between HNRNPA2B1 and immune cell infiltration levels were assessed using Spearman's correlation. Images of the results were obtained.

### 2.5. Investigation of the Enrichment of HNRNPA2B1-Associated Genes

HNRNPA2B1-binding proteins were explored using the STRING database (https://string-db.org/). Then, the top 100 HNRNPA2B1-related genes were investigated via “Similar Gene Detection” in GEPIA2. All the raw data were standardized using log2 TPM transformation. Finally, the selected genes were used for analysis based on the Kyoto Encyclopedia of Genes and Genomes (KEGG) pathway and Gene Ontology (GO) investigations.

### 2.6. Analysis of the Diagnostic Value

The pathological parameters of the tumor and normal tissue samples were obtained to evaluate the diagnostic value of HNRNPA2B1 by the receiver operating characteristic (ROC) curve via pROC and ggplot2 tools for investigation and visualization.

### 2.7. Gene Set Enrichment Analysis.

To assess the potential differences in biological functions between the high- and low-risk score subgroups, the gene set enrichment analysis (GSEA) software (https://www.gsea-msigdb.org/gsea/login.jsp) was used based on the hallmarks gene set (“h.all.v7.0.symbols.gmt”) as previously described.

## 3. Results

### 3.1. HNRNPA2B1 Levels and Location in Multiple Tumors

Using the Human Protein Atlas (HPA) database, normal tissues were examined for HNRNPA2B1 protein and RNA expression. HNRNPA2B1 proteins are found in the stomach, kidney, skin, liver, lung, and colon (Figure 1(a)). HNRNPA2B1 RNA levels were low in tongue tissues, whereas HNRNPA2B1 expression levels were high in lung tissues (Figure 1(b)). Furthermore, HNRNPA2B1 expression was found to be extremely high in cell lines (Figure 1(c)). The presence of HNRNPA2B1 in normal lung and cancer samples was investigated (Figures 1(d) and 1(e)). To further illustrate the intracellular locations of HNRNPA2B1, the distribution of HNRNPA2B1 within the nucleus and microtubules of A549 cells was examined via immunofluorescence labeling. It was revealed that HNRNPA2B1 colocalized with nuclear markers, implying that HNRNPA2B1 is subcellular localized in the nucleus. Conversely, HNRNPA2B1 showed no overlap with the microtubules (Figures 1(f) and 1(g)).

### 3.2. Induction of HNRNPA2B1 Levels in Different Cancer Types

In this study, the HNRNPA2B1 levels were explored in pan-cancer. The HNRNPA2B1 levels in different tumor samples were higher than the matching normal samples, including bladder urothelial carcinoma (BLCA), breast invasive carcinoma (BRCA), cholangiocarcinoma (CHOL), colon adenocarcinoma, esophageal carcinoma (ESCA), head and neck squamous cell carcinoma, liver hepatocellular carcinoma (LIHC), LUAD, lung squamous cell carcinoma (LUSC), rectum adenocarcinoma, and stomach adenocarcinoma (STAD) (Figures 2(a) and 2(b)). Data from the National Cancer Institute's Clinical Proteomic Tumor Analysis Consortium (CPTAC) database presented that there were higher HNRNPA2B1 protein levels in breast cancer, OC, colon cancer, and LUAD (Figure 2(c), *P* < 0.001).

The HEPIA2 dataset revealed an association of HNRNPA2B1 levels with the clinicopathological stages of adrenocortical carcinoma (ACC), but not with those of BLCA, BRCA, LUAD, LUSC, and OC (Figure 2(d)).

### 3.3. HNRNPA2B1 Prognostic Value in Pan-Cancer Based on TCGA Database

The Kaplan–Meier method was used to investigate HNRNPA2B1-related OS. HNRNPA2B1 levels have been associated with the survival rates of patients with cancer (Figure 3). Higher HNRNPA2B1 levels are associated with poor OS in LUAD (*P* = 0.00335), LGG (*P* = 4.1*e* − 05), KICH (*P* = 0.003), and ACC (*P* = 0.00053) (Figure 3(a)). Nonetheless, higher HNRNPA2B1 levels were associated with a poor THYM OS (*P* = 0.0018) (Figure 3(a)). Consistent with previous findings, HNRNPA2B1 expression levels in LUAD were significantly higher than that in control tissue samples, and the survival rate study revealed that higher HNRNPA2B1 levels are associated with a lower survival rate. Disease-free survival (DFS) study (Figure 3(b)) revealed an association between higher HNRNPA2B1 expression levels and poor DFS rates in ACC (*P* = 4.7*e* − 05), KICH (*P* = 0.043), LGG (*P* = 0.0012), LIHC (*P* = 0.043), and LUAD (*P* = 0.012). Furthermore, lower HNRNPA2B1 levels were associated with a poor DFS prognosis rate in THCA (*P* = 0.0045).

### 3.4. Interrelationships among HNRNPA2B1 Mutation, Hypomethylation, and Prognosis in LUAD

After confirming the prognostic significance of HNRNPA2B1, the cBioPortal tool was used to evaluate HNRNPA2B1 levels and mutations in LUAD. Patients with lung cancer had a higher mutation degree and number of mutation locations in HNRNPA2B1 (Figures 4(a)–4(c)). However, genetic changes in HNRNPA2B1 were not associated with lung cancer survival (Figure 4(d)). Based on the data presented above, it is reasonable to conclude that the genetic mutation of HNRNPA2B1 has no effect on the prognosis of patients with lung cancer. In addition, HNRNPA2B1 gene copy numbers and levels were analyzed using cBioPortal, and HNRNPA2B1 levels were found to be associated with gene copy numbers in LUAD (Figure 4(e)). Furthermore, analysis using the MethSurv tool revealed that patients with higher HNRNPA2B1 methylation levels had a worse OS than those with lower HNRNPA2B1 methylation levels. CpG sites, including cg19062098, located on the CpG island also revealed a poor prognosis (Figure 4(f)). The methylation status of HNRNPA2B1 in LUAD analyzed by the MethSurv tool is presented in Figure 4(g).

### 3.5. Protein Phosphorylation Evaluation Data

The HNRNPA2B1 phosphorylation levels between primary tumor tissues and normal tissue samples were examined using the CPTAC database. The HNRNPA2B1 phosphorylation sites in breast cancer (Figure 5(a)), OC (Figure 5(b)), and LUAD (Figure 5(c)) were investigated.

### 3.6. Association between HNRNPA2B1 Levels and Infiltration of Immune Cells in LUAD

TIMER was used to investigate the relationship between HNRNPA2B1 and immune cell or Treg cell infiltration. It showed a positive relationship between HNRNPA2B1 and cancer-linked fibroblast infiltration in ACC and LUAD, but a negative relationship in STAD (Figure 6(a)). HNRNPA2B1 levels in LUAD were found to be positively associated with cancer-linked fibroblast infiltration (Figure 6(a), Rho = 0.238, *P* = 8.52*e* − 08). It also revealed a positive association between HNRNPA2B1 levels and the extent of Treg cell infiltration in LIHC, UVM, and LUAD (Figure 6(b)). Here, HNRNPA2B1 levels in LUAD were positively associated with the extent of infiltration of Treg cells (Figure 6(b), Rho = 0.24, *P* = 7.06*e* − 08).

### 3.7. Enrichment Study of HNRNPA2B1-Related Partners

To determine the mechanism of HNRNPA2B1 in LUAD, the HNRNPA2B1-binding proteins and HNRNPA2B1-associated genes were assessed via the STRING and GEPIA2 websites. The top 100 experimentally validated proteins that bind to HNRNPA2B1 were attained via the STRING tool, and an interaction network was created (Figure 7(a)). Then, the top 100 HNRNPA2B1 correlation genes were selected via the GEPIA2, and we presented the connection between the top six genes and HNRNPA2B1 in pan-cancer and lung cancer (Figures 7(b) and 7(c)). The HNRNPA2B1 levels were positively associated with TAR DNA binding protein (TARDBP) (*R* = 0.82), DExH-Box Helicase 9 (DHX9) (*R* = 0.8), heterogeneous nuclear ribonucleoprotein R (HNRNPR) (*R* = 0.8), serine and arginine-rich splicing factor 1 (SRSF1) (*R* = 0.79), heterogeneous nuclear ribonucleoprotein D (HNRNPD) (*R* = 0.77), and heterogeneous nuclear ribonucleoprotein M (HNRNPM) (*R* = 0.76) genes (all *P* < 0.001) in pan-cancer. The HNRNPA2B1 levels were positively associated with TARDBP (*R* = 0.83), DHX9 (*R* = 0.73), HNRNPR (*R* = 0.77), SRSF1 (*R* = 0.79), HNRNPD (*R* = 0.75), and HNRNPM (*R* = 0.78) genes in lung cancer (Figure 7(c); all *P* < 0.001). Furthermore, an intersection analysis of HNRNPA2B1-binding proteins and the associated genes displayed 19 common partners (Figure 7(d)). Then, the KEGG enrichment investigation indicated that HNRNPA2B1 participates in the pathways associated with spliceosome, mRNA surveillance, and RNA degradation in cancers. Importantly, the effect of HNRNPA2B1 on pan-cancers may be connected with the cell cycle pathway (Figure 7(e)). The GO investigation revealed that RNA splicing, snRNA binding, and helicase activity were enriched (Figure 7(f)).

### 3.8. Diagnostic Value of HNRNPA2B1 Expression in Pan-Cancer

The ROC curve was used to explore the diagnostic value of HNRNPA2B1. It revealed that HNRNPA2B1 levels have potent diagnostic value for LUAD (AUC value = 0.837), LUSC (AUC value = 0.912), BRCA (AUC value = 0.883), ESCA (AUC value = 0.927), LIHC (AUC value = 0.931), and STAD (AUC value = 0.944) (Figure 8).

### 3.9. Gene Set Enrichment Analysis

GSEA was used to further investigate the molecular mechanism. The mitotic-spindle pathway was revealed to be the most relevant enrichment pathway in LUAD (Figure 9).

## 4. Discussion

Cancer is one of the major causes of patient death worldwide. Moreover, the rapid increase in cancer incidence and the attendant mortality called for new and more efficient treatment approaches [20, 21]. Recently, a few studies have described the association between HNRNPA2B1 and diseases, especially cancer [22–25]. Whether HNRNPA2B1 plays a key role in various cancer types remains unclear. Thus, this study assessed whether HNRNPA2B1 levels are associated with genetic alterations and immune cell infiltration in pan-cancer.

In a previous study, patients with oral squamous cell carcinoma who had higher HNRNPA2B1 expression had a poor prognosis [26]. Using the TIMER and GEPIA2 tools, we found that HNRNPA2B1 is present in abnormally high levels in various tumor types, such as breast cancer, OC, and LUAD. HNRNPA2B1 overexpression is associated with a poor prognosis according to the Kaplan–Meier curve. We found that high HNRNPA2B1 levels were associated with a poor prognosis of ACC, KICH, LGG, and LUAD in pan-cancer studies. As a result, more research into the roles and mechanisms of action of HNRNPA2B1 in the aforementioned cancer types is required. This study reports that HNRNPA2B1 may affect various mechanisms that contribute to cancer development. Using the cBioPortal database, the mutation analysis revealed that BLCA has the highest frequency of missense mutations, while esophageal adenocarcinoma has the highest frequency of amplification mutations. Furthermore, HNRNPA2B1 mutations did not affect OS or DFS in LUAD. HNRNPA2B1 genetic and epigenetic changes influence cancer progression regulation.

The phosphorylated HNRNPA2B1 levels were evaluated in breast cancer, OC, and LUAD. It revealed that the phosphorylation of HNRNPA2B1 presented an increasing pattern in these cancer types. Nonetheless, the association of alterations in the phosphorylation status of HNRNPA2B1 has not been clarified, and further assessments are necessary to investigate this hypothesis.

The immune microenvironment, especially the immune cells, is widely known to be involved in cancer development and elimination [27–30]. The current findings further suggested an association between HNRNPA2B1 and the infiltration of cancer-linked fibroblasts or Treg cells in different cancer types. Whether HNRNPA2B1 acts as an oncogene via regulation of the immune microenvironment still needs to be elucidated.

Lastly, the present study facilitated the effect of HNRNPA2B1 on pan-cancers by GO and KEGG evaluations, and our results revealed that HNRNPA2B1 plays a key role in spliceosome- and cell cycle-related pathways. Nevertheless, the association between HNRNPA2B1 and the cell cycle remains unknown. Thus, further experiments are necessary to verify the relationship between HNRNPA2B1 and the cell cycle.

GSEA was used to further investigate the molecular mechanism. The mitotic-spindle pathway was discovered to be the most relevant enrichment pathway in LUAD. As a result, it will be necessary to investigate the signal in a future study to better understand this phenomenon. The advancement of interaction prediction research in various fields of computational biology would provide valuable insights into genetic markers and ncRNAs related to different cancers, such as miRNA–lncRNA interaction prediction [31–34]. It has been found that HNRNPA2B1 serves as a lncRNA- or miRNA-binding protein; therefore, additional research is needed to explore the relationship between HNRNPA2B1 and miRNA–lncRNA interaction.

## 5. Conclusions

Overall, this pan-cancer analysis of HNRNPA2B1 revealed that HNRNPA2B1 overexpression is associated with changes in immune cell infiltration, spliceosome, and cell cycle signaling, as well as patient prognosis in various tumors. As a result, HNRNPA2B1 may function as a potential promoter and biomarker in the development and prognosis of cancer. This study adds to our understanding of the importance of HNRNPA2B1 functions in various tumors.

## Figures and Tables

**Figure 1:** HNRNPA2B1 expression and location. (a) HNRNPA2B1 protein level results in the normal tissues. (b) HNRNPA2B1 RNA level results in the normal tissues. (c) HNRNPA2B1 level results in the cell line. (d, e) HNRNPA2B1 location in lung cancer was gained from the Human Protein Atlas; (f) HNRNPA2B1 is positioned in the nucleus; (g) HNRNPA2B1 is located in A549 cell nucleus, the nucleus staining is presented in blue, and the HNRNPA2B1 protein staining is presented in green.

**Figure 2:** HNRNPA2B1 level in tumors and normal tissues. (a) HNRNPA2B1 level in tumors samples and the unpaired normal tissues. (b) HNRNPA2B1 level in the tumors and the paired adjacent normal tissues. (c) HNRNPA2B1 protein level in the tumors and the normal tissues using CPTAC. (d) The relationship between HNRNPA2B1 level and the pathological stages of tumor.

**Figure 3:** Association between HNRNPA2B1 level and cancers prognosis. The Kaplan–Meier curves of overall survival and disease-free survival investigate differences with high/low HNRNPA2B1 levels from TCGA database.

**Figure 4:** Mutation characteristic of HNRNPA2B1 in pan-cancer. The alteration occurrence with mutation form (a) and mutation location (b, c) are demonstrated using the cBioPortal. (d) The possible connection between mutation pattern and overall and disease-free survival of lung cancer was evaluated. (e) Relationships between HNRNPA2B1 level and copy number. (f) The Kaplan–Meier survival of the promoter methylation of HNRNPA2B1 in LUAD. (g) The methylation level of HNRNPA2B1 is imagined in LUAD.

**Figure 5:** Phosphorylation levels of HNRNPA2B1 in breast cancer, ovarian cancer, and lung adenocarcinoma and the relationship with gene expression.

**Figure 6:** HNRNPA2B1 level and immune infiltration. (a) Relationship of HNRNPA2B1 level with cancer-linked fibroblasts levels in ACC, LUAD, and STAD. (b) The possible association between HNRNPA2B1 level and the infiltration level of Treg cells in LIHC, LUAD and UVM.

**Figure 7:** HNRNPA2B1-related gene enrichment analysis. (a) HNRNPA2B1-binding proteins (top 100) attained using the STRING approach. (b) The top 6 HNRNPA2B1-linked genes were gained from TCGA and investigated the level association between HNRNPA2B1 and the targeting genes in pan-cancer by the GEPIA2. (c) The top 6 HNRNPA2B1-linked genes were gained from TCGA and investigated the level association between HNRNPA2B1 and the targeting genes in lung cancer by the GEPIA2. (d) A crossing study of HNRNPA2B1-binding proteins and HNRNPA2B1-correlated genes. (e) KEGG analysis of the HNRNPA2B1-binding proteins and HNRNPA2B1-correlated genes. (f) GO analysis of the HNRNPA2B1-binding proteins and HNRNPA2B1-correlated genes.

**Figure 8:** Receiver operating characteristic curve for HNRNPA2B1 level in different cancer.

**Figure 9:** GSEA data indicated the most relevant enrichment signal.

## Data Availability

The data analyzed during the current study are available from the corresponding author on reasonable request.
